The article "Aux/IAA Gene Family in Plants: Molecular Structure, Regulation, and Function" was published in 2018. Journal: Int J Mol Sci.

# *Aux/IAA* Gene Family in Plants: Molecular Structure, Regulation, and Function

**DOI:** 10.3390/ijms19010259

**Published:** 2018-01-16

**Authors:** Jie Luo, Jing-Jing Zhou, Jin-Zhi Zhang

**Affiliations:** 1 College of Horticulture and Forestry Science, Hubei Engineering Technology Research Center for Forestry Information, Huazhong Agricultural University, Wuhan 430070, China; luojie@mail.hzau.edu.cn; 2 Key Laboratory of Horticultural Plant Biology (Ministry of Education), College of Horticulture and Forestry Science, Huazhong Agricultural University, Wuhan 430070, China

**Keywords:** auxin, *Aux*/*IAA* gene family, regulation, function

## Abstract

Auxin plays a crucial role in the diverse cellular and developmental responses of plants across their lifespan. Plants can quickly sense and respond to changes in auxin levels, and these responses involve several major classes of auxin-responsive genes, including the *Auxin/Indole-3-Acetic Acid* (*Aux/IAA*) family, the *auxin response factor* (*ARF*) family, *small auxin upregulated RNA* (*SAUR*), and the *auxin-responsive Gretchen Hagen3* (*GH3*) family. Aux/IAA proteins are short-lived nuclear proteins comprising several highly conserved domains that are encoded by the auxin early response gene family. These proteins have specific domains that interact with ARFs and inhibit the transcription of genes activated by ARFs. Molecular studies have revealed that Aux/IAA family members can form diverse dimers with *ARFs* to regulate genes in various ways. Functional analyses of Aux/IAA family members have indicated that they have various roles in plant development, such as root development, shoot growth, and fruit ripening. In this review, recently discovered details regarding the molecular characteristics, regulation, and protein–protein interactions of the Aux/IAA proteins are discussed. These details provide new insights into the molecular basis of the Aux/IAA protein functions in plant developmental processes.

## 1. Introduction

In plants, many developmental processes are finely tuned by auxin, such as vascular tissue formation, adventitious root initiation, tropistic responses, apical dominance, and flower and fruit development. Auxin also affects cellular processes, such as cell division, enlargement, and differentiation [1,2,3,4]. Dynamic spatial and temporal changes in auxin levels can trigger gene reprogramming precisely and rapidly, which requires auxin early response genes, such as the Auxin/Indole-3-Acetic Acid (Aux/IAA) family, the auxin response factor (ARF) family, small auxin upregulated RNA (SAUR), aminocyclopropane-1-carboxylic acid synthase (ACS), glutathione-*S*-transferase (GH2/4-like), and the auxin-responsive Gretchen Hagen3 (GH3) family [3,5,6]. Among these genes, Aux/IAA family members have been identified as short-lived nuclear proteins that play a crucial role in repressing the expression levels of genes activated by ARFs [7,8]. It has also been demonstrated that auxin-mediated transcriptional regulation is exclusively dependent on the functions of Aux/IAA [9]. Aux/IAA proteins have been suggested to bind with ARFs and prevent activation of auxin-responsive genes in the absence of auxin. At high auxin levels, these proteins can be ubiquitinated by interacting with TRANSPORT INHIBITOR RESPONSE 1/AUXIN SIGNALING F-BOX (TIR1/AFB) receptors and subsequently degraded via the 26S proteasome [10,11,12]. The released ARFs regulate the expression of auxin-responsive genes [10]. The different TIR1/AFB-Aux/IAA protein combinations usually have differential auxin-binding affinities, and the auxin levels are different in different tissues and developmental phases, which results in distinct auxin-sensing effects [9,11,13,14]. Thus, the spatial–temporal dynamic change in auxin levels can be finely transformed into gene reprogramming signaling, thereby regulating the processes of plant growth and development in a precise manner.

The article "Aux/IAA Gene Family in Plants: Molecular Structure, Regulation, and Function" was published in 2018. Journal: Int J Mol Sci.

Over the past two decades, mutations in *Aux*/*IAA* genes have been intensely studied in *Arabidopsis*, and these studies have revealed that the members of this family display distinct functions in plant growth and development processes [15,16,17,18]. To date, 29 *Aux*/*IAA* gene family members in *Arabidopsis* have been isolated [18,19,20]. Meanwhile, many candidate genes that potentially regulate the stability of Aux/IAA proteins have also been identified [21,22]. It is noteworthy that a large number of Aux/IAA family members have also been identified in other plants, including *Eucalyptus grandis*, *Solanum lycopersicon*, *Cucumis sativus*, *Populus trichocarpa*, *Zea mays*, and *Oryza sativa* [23,24,25,26,27,28,29]. Recently, through the combined application of physiological, genetic, molecular, and biochemical methods, increasingly abundant new information regarding the mechanisms of Aux/IAA in regulating auxin signal transduction and auxin degradation has been obtained, and this information provides valuable opportunities to clarify the developmental processes fine-tuned by auxin signaling in plants. In this review, recent advances in the roles of Aux/IAA in regulating plant growth and development, as well as global and new insights into the underlying molecular mechanisms of these processes, will be presented. 

## 2. Identification, Gene Duplication, and Molecular Structure of Aux/IAA Proteins in Plants

The first isolated *Aux*/*IAA* genes were the *PS-IAA4*/*5* and *PS-IAA6* genes from pea [30,31]. Subsequently, 14 Aux/IAA genes were isolated from *Arabidopsis* based on the homologues to *PS-IAA4/5* and *PS-IAA6* [6]. With the advent of genome sequencing, the IAA/Aux gene family has been identified in 30 plant species by genome-wide analysis, including 29 genes from *Arabidopsis*, 55 from *Brassica rapa*, 26 from Citrus, 26 from *Eucalyptus grandis*, 26 from *Solanum lycopersicum*, 26 from *Solanum tuberosum*, 26 from *Vitis vinifera*, and 35 from *Populus trichocarpa* (Table 1) [19,23,24,26,32,33,34,35]. Among these species, the largest Aux/IAA gene family (119 members) was observed in the genome of *Brassica napus*, largely as a result of duplication in different subgenomes [36]. In addition, a large proportion of Aux/IAA genes was observed to be generated from gene duplication events during the course of evolution, such as segmental duplication, tandem duplication, or both [29,37]. For example, 76% and 90% of *Aux*/*IAA* genes were segmentally duplicated in the genomes of *Arabidopsis* and *Glycine max*, respectively [29,37]. Curiously, only 6% (2 out of 31) of *Aux*/*IAA* genes were tandemly correlated in *Picea abies* [29], even though this species has undergone numerous duplications [38]. The duplication events of the *Aux*/*IAA* gene family seem to coincide with whole-genome duplication (WGD) [29,37]. For instance, two WGD events and one whole-gene triplication (WGT) have been found in the genome of *Glycine max*, but no WGD event was observed during the genome evolution of *Picea abies* [37,38,39]. Compared with higher-order plants, no or fewer Aux/IAA genes were identified in lower plants, such as *Chlamydomonas reinhardtii* (0), *Marchantia polymorpha* (1), *Physcomitrella patens* (3), and *Selaginella moellendorffii* (9) [29,40,41,42]. Thus, the expanded *Aux*/*IAA* gene members in land plants create functional redundancy and may be associated with new functions to adapt to environmental changes [43,44,45].

The article "Aux/IAA Gene Family in Plants: Molecular Structure, Regulation, and Function" was published in 2018. Journal: Int J Mol Sci.

Bioinformatic and molecular studies have relabeled most Aux/IAA proteins to indicate that they generally harbor four conserved characteristic domains: Domain I, II, III, and IV (Figure 1) [51]. Domain I has been identified as a repression domain bearing an ethylene response factor (ERF)–associated amphiphilic repression (EAR) motif, “LxLxL”, which can recruit a TOPLESS (TPL) co-repressor [52]. Domain II is the auxin degron with a conserved “GWPPV” motif, which can directly interact with SCF^TIR1^ and plays a role in rapid protein turnover [32,53]. Domain II also contains a bipartite structural nuclear localization signal (NLS) with the invariant basic doublet KR [6]. Recently, a conserved lysine–arginine (KR) motif located between the ERF-EAR motif and Domain II was identified as a rate motif that aids in tuning the dynamic turnover of Aux/IAA proteins [54,55]. More recently, flexible hotspots with certain specific lysine residues have been identified in the degron-flanking regions, which are closely linked to ubiquitylation mediated by TIR1 [56]. Domain III contains an amphipathic βαα-fold with a structure and function similar to the DNA recognition motif in Arc and MetJ repressors [7,57]. Further studies confirmed the roles of the βαα-fold in homo- and heterodimerization with Aux/IAA and/or ARF proteins [51,57,58]. Domain IV comprises an acidic region and an SV40 type NLS (PKKKRKV) [59]. In addition, a conserved “GDVP” motif between β4 and α2 in Domain IV may contribute to electrostatic protein interactions [59]. Domain III and IV (namely, Domain III/IV) share homology with the carboxy-terminal dimerization domain (CTD) in ARF proteins, which is involved in regulating ARF activity by interacting with Aux/IAA and ARF family proteins via the type I/II Phox and Bem1p (PB1) protein–protein interaction domain [51,58,59,60]. The type I/II PB1 domains share both an acidic motif (type I) and basic motif (type II), and the type I motif contains the conserved octicosapeptide (OPCA)-like motif (Dx(D/E)GDx8[E/D], the Phox and Cdc motif, and the atypical protein kinase C interaction domain motif [59,61]. These identified motifs provide physical binding sites for regulating the auxin signaling pathway.

Although most Aux/IAA proteins harbor the typical four domains, a considerable number of truncated Aux/IAA proteins have also been found in different plant species (Table 1). For instance, two Aux/IAA proteins (AtIAA29 and AtIAA33) in *Arabidopsis*, three Aux/IAA proteins (SlIAA13, SlIAA16, and SlIAA20) in tomato, and five Aux/IAA proteins (StIAA13, StIAA15, StIAA16, StIAA18, and StIAA20) in potato lack Domains I and II [29,34]. Meanwhile, some truncated proteins without Domain III or IV have been identified, such as CpIAA11, CpIAA19, CpIAA27, and CpIAA31 from *Carica papaya* [47]. Additionally, a large proportion of truncated Aux/IAA proteins have been found in *Amborella trichopoda*, *Cicer arietinum*, *Phalaenopsis equestris*, *Picea abies*, *Selaginella moellendorffii*, and *Triticum aestivum* (Table 1) [29,37,40,50]. In addition to lacking some essential domains, a tandem duplication of domain II was exclusively identified in PoptrIAA7.1 (a homolog of *Arabidopsis IAA7*) and conserved only in *Populus* species [26]. Overall, the variations in these domains may contribute to the diverse functions in the auxin signaling pathway, which further facilitate the multiple roles played by Aux/IAA in response to changes in the environment among plants.

The article "Aux/IAA Gene Family in Plants: Molecular Structure, Regulation, and Function" was published in 2018. Journal: Int J Mol Sci.

## 3. Interaction of Aux/IAA Proteins in Plants

Plants can sense and respond to auxin signaling in a precise and rapid manner, and this response involves a group of genes called the early auxin response genes [44]. The Aux/IAA proteins are well-known as the early auxin response proteins and participate in auxin signaling through interacting with ARF proteins as transcriptional repressors [7,9,62]. The functions of Aux/IAA proteins in auxin signaling have been well summarized [63,64]. In brief, Aux/IAA and ARF have the same type I/II PB1 domain in their homologues, Domain III/IV, and the type I/II PB1 domain carries both positive and negative charges, which facilitate head-to-tail homo- and heterodimerization of Aux/IAA and ARF via electrostatic interactions [58,61,65,66]. At low auxin levels, Aux/IAA proteins directly dimerize with ARF proteins to prevent their physical interaction with transcription initiation complexes and recruit TPL/TPR co-repressors in the EAR domain [52,67]. The recruited TPL/TPR proteins interact with histone deacetylases to induce chromatin condensation [52]. At high auxin levels, the Aux/IAA proteins are brought together with TIR1/AFB proteins by auxin. The F-box in TIR1/AFB proteins can be recognized by SCF-type ubiquitin protein ligase complexes, and subsequently, the Aux/IAA proteins are poly-ubiquitinated by SCF proteins and degraded through the 26S proteasome proteolytic pathway [12,63,64]. Next, the released ARF proteins may recruit SWITCH/SUCROSE NONFERMENTING (SWI/SNF) to remodel the chromatin into an active state and bind to the auxin response DNA *cis*-elements (AuxREs) to trigger changes in their target auxin response genes at the transcriptional level [5,62]. Based on this mechanism, auxin signaling can result in changes in gene expression levels.

The interaction and regulation of Aux/IAA proteins are closely associated with their modular structure. Domains I and II are well known for their roles in stabilizing Aux/IAA proteins, and Domain II contains a GWPP-core degron sequence, which is the core binding site with TIR/AFB proteins and auxin [68]. Crystal structures have shown that the leucine-rich repeat (LRR) domain of TIR/AFB proteins can form an auxin binding pocket, which allows auxin to anchor at the bottom and “glue” its “GWPP” motif in the degron of Aux/IAA proteins and to occupy the rest of the area of this pocket [12]. Thus, even single-point mutations in the degron region reduce the affinity to TIR/AFB proteins and hamper the degradation of Aux/IAA proteins [69]. In addition, the conserved rate motif, KR, also facilitates the turnover of Aux/IAA proteins, and plants without this rate motif exhibit insensitive auxin response phenotypes similar to plants with degron mutations [54]. Recent evidence showed that auxin can regulate the 26S proteasome-mediated degradation of ubiquitinated Aux/IAA by remobilizing PROTEASOME REGULATOR1 (PTRE1) from the nucleus to the plasma membrane [70,71]. The degradation rates and ubiquitination sites are varied among Aux/IAA proteins, and lysine residues are not necessary for degradation [72]. Variations in the ubiquitylation sites in flexible hotspots of the degron-flanking regions also lead to distinct auxin affinities, which correspond to the degradation dynamics among different IAA proteins [56]. The negative feedback regulation of 26S proteasome activity may contribute to avoiding over-enhancement of auxin signaling and excessive degradation of Aux/IAA proteins [70]. In addition to Domains I and II, Domains III and IV, which are homologous to the carboxy-terminal dimerization domain (CTD) of ARFs, contain the well-known PB1 domain [61]. Based on thermodynamic and structural approaches, a two-pronged electrostatic interaction was identified in the PB1 domain, and the roles of the charged residues on the basic and acidic faces in stabilizing the protein–protein interaction have been revealed [60]. Although Aux/IAA and ARF can form homo- or hetero-oligomers via their PB1 domains, case studies of ARF5 and IAA17 have revealed that their hetero-oligomers have up to 100-fold greater affinity than their homo-oligomers [73]. These studies shed new light on how these PB1-containing proteins interact with each other at the atomic level to facilitate auxin signaling.

The article "Aux/IAA Gene Family in Plants: Molecular Structure, Regulation, and Function" was published in 2018. Journal: Int J Mol Sci.

Based on large-scale interactome analyses conducted in *Arabidopsis* using affinity capture-Western/MS, yeast two-hybrid, reconstituted complex, and protein-fragment complementation assay (PCA) approaches, a comprehensive physical interactome map of Aux/IAA proteins has been developed in recent years (Figure 2) [13,17,20,74]. This interactome map consists of the essential auxin signaling transduction components mediated by Aux/IAA proteins (Figure 2). For instance, 29 Aux/IAA proteins had physical contact with 20 ARF proteins via 544 interactions, and Aux/IAA homo-interactions and Aux/IAA-ARF hetero-interactions occupied 47% and 45% of interactions, respectively (Figure 2). All 29 Aux/IAA proteins interacted with each other with 253 interactions, and only 13 ARF shared 22 homo-interactions (Figure 2). TPL/TPR proteins are co-repressors that bind to the EAR domain of Aux/IAA. In the interaction network, four TPL/TPR proteins were identified, and most Aux/IAA proteins had physical interactions with these four TPL/TPR proteins, except IAA5, IAA6, IAA9, IAA14, IAA15, IAA20, IAA29, IAA30, IAA31, IAA32, IAA33, and IAA34 (Figure 2). Recently, a report demonstrated that the homo-oligomerization of TIR1 in *Arabidopsis* was another pathway for regulating auxin signaling by affecting Aux/IAA protein turnover [75]. In the interactome map, four out of six TIR1/AFB proteins were involved in this interactome, but only 11 Aux/IAA proteins had direct physical interactions with the four TIR1/AFB proteins (Figure 2). Thus, the large number of homo-interactions among Aux/IAA proteins and the lack of physical interaction with the TIR1/AFB proteins imply that many Aux/IAA proteins may only function as heterodimerization partners and may not participate in ubiquitination and turnover processes. It should also be noted that most interactions in the Aux/IAA interactome map come from in vitro experiments, and the specific roles of these interactions in auxin signaling need to be further verified with in vivo evidence. These identified essential components, as well as potential protein interactors in the Aux/IAA-mediating auxin signaling pathway, provide comprehensive maps of how changes in auxin levels are reflected in gene reprogramming events.

The article "Aux/IAA Gene Family in Plants: Molecular Structure, Regulation, and Function" was published in 2018. Journal: Int J Mol Sci.

## 4. Aux/IAA Proteins Might be Regulated at Different Levels

In addition to interacting with the auxin signaling components, several interesting transcription factors and signaling proteins that potentially interact with Aux/IAA have been identified (Figure 3) [79]. A recent study showed that RGA-LIKE3 (RGL3) competitively interacted with IAA17 to protect IAA17 from TIR1, and the interaction between these two proteins enhanced the nitric oxide (NO)-mediated salt stress response [80]. Meanwhile, NO donors also increase auxin-dependent gene expression, while NO depletion blocks Aux/IAA protein degradation [81]. Additionally, *S*-nitrosylation of TIR1 at the post-translational level reinforced the TIR1–Aux/IAA interaction and facilitated the turnover of Aux/IAA proteins [81]. Further study has found that a set of spatially clustered residues in TIR1 guide their oligomerization in *Arabidopsis*, and this process is required for IAA protein turnover and auxin signaling transduction [75]. Interestingly, mutations in the identified amino acid residues for *S*-nitrosylation also hamper TIR1 oligomerization, which implies that NO may affect TIR1 oligomerization to regulate auxin signaling [75]. During *Arabidopsis* root development, it was reported that an E2 enzyme for Lys63-linked ubiquitination (UBC13) can regulate the stability of Aux/IAA to control auxin-mediated root development, and this process may be involved in suppressing the activity of the SCF^TIR1^ complex [82]. These data suggest that regulation of the stability of Aux/IAA proteins by other factors plays crucial roles in mediating the auxin signaling pathway in plants. A chromatin-remodeling factor, PICKLE (PKL), was shown to be essential for IAA17-mediated repression of ARF7/19 activity and for lateral root initiation [83]. In addition, *IAA3* has been shown to be a target of two different histone acetyltransferases, specifically, auxin influx carrier LIKE AUXIN RESISTANT 2 (LAX2) and general control nonderepressible 5 (GCN5), which indicates that the *Aux*/*IAA* genes can also be regulated by epigenetic modifications [84,85]. Thus, the epigenetic modifications also play an important role in regulating the expression levels of *Aux*/*IAA* genes. Furthermore, the transcription factor PHYTOCHROME INTERACTING FACTOR 4 (PIF4) can promote the expression level of *IAA19* and *IAA29* by directly binding to their promoters to repress the activity of ARF7, thereby negatively regulating phototropism and auxin signaling [86]. Recent studies have uncovered that 21 of 29 *Aux*/*IAA* genes are the targets of three PIFs (PIF3, PIF4, and PIF5), and 12 *Aux*/*IAA* genes are upregulated in response to natural shade [87,88]. These results highlight the crucial roles of *Aux/IAA* genes in auxin-mediated light responses. Another transcription factor, *MYB77*, had in vitro interactions with ARF7 or IAA19 to control lateral root formation [74,89]. In addition, IAA29 can competitively interact with WRKY57 to antagonize jasmonic acid-induced leaf senescence [90,91]. Recently, other stress-related transcription factors, such as the dehydration-responsive element binding proteins (DREB1)/C-repeat (CRT) binding factor (CBF) family, have been shown to directly bind to the promoters of *IAAs* [92]. For instance, CBF1 and DREB2A can directly regulate the transcription level of *IAA5* and *IAA19*; the latter genes are essential for overcoming desiccation stress in *Arabidopsis* [92]. The basic leucine zipper (bZIP) transcription factor bZIP11 balances energy homeostasis and primary root growth by directly activating the transcriptional reprogramming of *IAA3*, which is a suppressor of root growth [93]. In addition, a nuclear import receptor IMPORTIN-ALPHA 6 (IMPα6) can efficiently take up IAA12 into the nucleus, and this process is required for maintaining enough short-lived IAA12 in the nucleus to regulate primary root initiation [94]. In rice, an inositol polyphosphate kinase (OsIPK2) stabilized OsIAA11 protein by interacting with its Domain II, and overexpression of OsIPK2 caused typical auxin insensitivity and failure to form the lateral root [95]. OsCYP2 (a cyclophilin gene) directly interacts with its co-chaperone suppressor of the G2 allele of skp1 (OsSGT1) to regulate lateral root initiation by promoting the turnover of Aux/IAA proteins [96]. Further study identified a C2HC-type zinc finger protein (OsZFP) that can directly interact with OsCYP2 to regulate lateral root development via the IAA pathway, and *OsIAA23* might participate in this *OsZFP*-mediated auxin signaling process [97]. Interestingly, the capsid protein P2 from the rice dwarf virus (RDV) can directly interact with OsIAA10 and block the degradation processes mediated by OsTIR1, and mutations in *OsIAA10* enhanced rice resistance to this virus [98]. 

The article "Aux/IAA Gene Family in Plants: Molecular Structure, Regulation, and Function" was published in 2018. Journal: Int J Mol Sci.

Meanwhile, post-translational modifications also play crucial roles in regulating Aux/IAA proteins (Figure 3) [99]. For instance, previous experiments verified that IAA1, IAA3, IAA9, and IAA17 of *Arabidopsis* can be phosphorylated by PHYTOCHROME A (PHYA) in vitro, which provides evidence of auxin involvement in light signaling [100]. In another recent paper, a cyclophilin-type peptidyl-prolyl *cis*/*trans* isomerase, LATERAL ROOTLESS2 (LRT2), was shown to catalyze the peptidyl-prolyl isomerization of OsIAA11, which facilitates OsIAA11-OsTIR1 interactions and the turnover of OsIAA11 via the 26S proteasome [101]. Recently, a large number of microRNAs (miRNAs) have also been shown to target the upstream regulators of Aux/IAA, but information on posttranscriptional regulation of Aux/IAA proteins by miRNA is still very limited [9,102]. The first miRNA found to cleave *Aux/IAA* has been identified in *Arabidopsis*, and this miRNA, *miR847*, targets *IAA28* mRNA for degradation and positively regulates lateral organ development as a positive regulator [103]. However, the information about post-translational regulation of Aux/IAA proteins is still very limited; further studies are needed to shed new light on this area.

## 5. Functional Roles of Aux/IAA Genes during Plant Growth and Development Processes

Although there are 29 Aux/IAA proteins in *Arabidopsis* (with some functional redundancy), most mutations in Aux/IAA proteins display similar phenotypes in which auxin signaling transduction is hampered, leading to defects in diverse developmental processes such as embryo development, lateral root initiation and elongation, hypocotyl growth, tropisms, flower organ development, and other processes (Figure 4) [17,18,19]. For example, a gain-of-function mutant, *iaa1*/*axr5*, showed defects in root and shoot tropisms [104], but gain-of-function mutations in *iaa2* and *iaa6* lead to similar phenotypes, which exhibited a short hypocotyl and upcurled leaves, in *Arabidopsis* [15,105]. IAA3, IAA14, and IAA18 act redundantly in controlling lateral root formation by interacting with two ARF proteins (ARF7 and ARF19). Additionally, phenotypic analysis of transgenic *Arabidopsis* variants differing in the IAA14 degradation rate indicated that the timing of lateral root initiation is finely tuned by the turnover rate of IAA14 [106]. *IAA7*/*AXR2* controls the morphological responses induced by light, such as inhibiting hypocotyl elongation and promoting leaf development, as observed in *iaa7/axr2-1* mutants cultured in the dark [107]. IAA8 can interact with TIR1 to regulate lateral root formation, and overexpression of this gene caused abnormal gravitropism [108]. A mutation in domain II of *IAA8* resulted in abnormal flower organs with low jasmonic acid levels, which was mediated by its interactions with *ARF6* and *AFR8* [17,109]. IAA12 regulates root meristem initiation during early embryogenesis by interacting with the ARF5 protein, the latter of which is essential for embryonic root and embryo patterning [110,111]. Stabilized *iaa16* mutants display smaller rosettes, shorter root hairs, fewer lateral roots and shorter anther filament elongations than the wild type, and the homozygous *iaa16* mutants are not fertile [16]. *IAA17* is involved in some typical phenotypes controlled by auxin signaling, such as hypocotyl elongation, root gravitropism, and root hair and adventitious root formation [112,113]. A recent report showed that *IAA17* was also involved in cytosolic glutamine synthetase (*GLN1;2*)-mediated ammonium assimilation in *Arabidopsis* root [114]. A gain-of-function analysis verified the roles that *IAA18* plays in embryonic apical patterning by repressing the activity of ARF5 and other ARFs [115]. Interestingly, transcripts of *IAA18* and *IAA28* can be transported from mature leaves to the root via phloem to negatively regulate lateral root formation [116]. IAA19 participated in hypocotyl growth and lateral root formation by interacting with ARF7, and the *IAA19* mutant failed to maintain hypocotyl gravitropism and regular lateral roots [117]. Gain-of-function *iaa28-1* mutants show a strong auxin phenotype with failure to form lateral roots and a reduction in plant size and apical dominance [118]. Meanwhile, *IAA28* also participates in the process of lateral root founder cell identity by negatively regulating the activity of its downstream transcription factor, GATA23 [119]. Overexpression of three non-canonical *Aux/IAA* genes (*IAA20*, *IAA30*, and *IAA31*) results in similar aberrant phenotypes, and plants with *IAA20* overexpression show modified gravitropic root and hypocotyl growth and collapse of root apical meristem after germination [120].

The article "Aux/IAA Gene Family in Plants: Molecular Structure, Regulation, and Function" was published in 2018. Journal: Int J Mol Sci.

In addition to *Arabidopsis*, significant achievements have also been made in understanding the roles of Aux/IAA proteins in auxin signaling in other plants, such as tomato, potato, rice, and poplar [95,121,122,123,124]. In tomato, *SiIAA3* has been verified as a molecular bridge between auxin and ethylene signaling pathways, and *SiIAA3* RNAi plants display decreased petiole epinasty in light-grown seedlings and an exaggerated curvature of the apical hook under dark conditions [121]. *SiIAA9* controls multiple processes mediated by auxin signaling, such as apical dominance, leaf morphogenesis, flower organ development, and fruit set and development [125,126,127]. Mutations in *SiIAA9* lead to abnormal leaf shape and parthenocarpic fruits [125,126,127]. Recently, the CRISPR/Cas9 system was optimized to obtain *SlIAA9-crispr* in tomato plant (*Solanum lycopersicum*) mutants, which have phonotypes similar to *SiIAA9* mutant plants, e.g., abnormal leaves and parthenocarpy [128]. *SlIAA15* plays multiple roles during tomato developmental processes, and *SlIAA15-*suppressed plants exhibit enhanced lateral root formation, modified development of axillary shoots, decreased trichome number and fruit set, and increased leaf thickness [129]. *SiIAA17* plays crucial roles in controlling fruit quality, and *SiIAA17*-silenced lines display larger fruit with a thicker pericarp than the wild-type line [130]. *SiIAA27* RNAi plants display modified reproductive organ anatomy and reduced expression levels of genes involved in chlorophyll synthesis [131]. More recently, *SlIAA27* has been shown to positively regulate the formation of arbuscular mycorrhiza and participate in strigolactone biosynthesis by regulating the expression level of *NODULATION SIGNALING PATHWAY1* (*NSP1*) [132]. In potato, *StIAA2* repression results in altered shoot morphogenesis, increased plant height, and petiole hyponasty, and transcriptional reprogramming of other *StIAA* genes [122]. For members of the *Aux*/*IAA* gene family in rice, *OsIAA1* is induced by auxin and plays a role in light response and coleoptile elongation in rice [133]. Overexpression of *OsIAA4* in rice leads to less sensitivity to exogenous auxin, dwarfism, and more tiller angles in comparison with wild-type plants [134]. Overexpression of *OsIAA6* enhances tolerance to drought, however, loss-of-function mutants of *OsIAA6* display much more tiller outgrowth than does the wild type [135]. Conversely, overexpression of *OsIAA10* increases the number of tillers [98]. Degradation of OsIAA11 is essential for initiating lateral root formation, and mutations in the degron of OsIAA11 stabilize this protein and produce defects in the lateral root [95,96,136]. Gain-of-function *OsIAA13* mutants also display phenotypes of reduced lateral roots and defects in the gravitropic response, which are closely related to transcriptional reprograming of the set of genes involved in lateral root initiation [137]. *OsIAA23* is essential for postembryonic maintenance of the quiescent center by auxin signaling in rice [138]. In maize, IAA10 can repress the expression level of the *LATERAL ROOT PRIMORDIA 1* (*LRP1*) gene by directly binding to its promoter, and the gain-of-function mutant *iaa11* (*rum1*) cannot activate the expression of *LRP1* and fails to initiate seminal and lateral roots [139].

The article "Aux/IAA Gene Family in Plants: Molecular Structure, Regulation, and Function" was published in 2018. Journal: Int J Mol Sci.

In woody plants, overexpression of *PttIAA3m* causes global auxin-mediated gene reprogramming, which is closely linked to cambial cell division and secondary xylem development in hybrid aspen [123]. Overexpression of *PtrIAA14.1* (a homolog of *Arabidopsis IAA7*) in *Arabidopsis* confirms its roles in regulating vascular patterning via interaction with AFR5 [140]. Recently, another study verified the role of *Eucalyptus EgrIAA4* in fiber formation and secondary cell wall deposition by heterologous expression of this gene in *Arabidopsis* [23]. 

## 6. Conclusions and Perspectives

Over the last decade, remarkable progress has been made in understanding the mechanism of auxin perception and signaling transduction processes through forward and reverse genetic approaches. These advances reveal that *Aux*/*IAA* genes act as hub factors that regulate gene expression in auxin signaling transduction, and understanding of their molecular functions and regulatory machinery in plant growth and development has been greatly enhanced. However, concerning the processes of the *Aux*/*IAA*-mediated auxin signaling pathway, there are still many gaps that remain to be resolved. For example, there is still very limited information regarding the regulation of *Aux*/*IAA* genes at both transcriptional and post-transcriptional levels. Aux/IAA proteins have many interactions with other proteins in interactome maps, and the specific roles of these interactions are largely unknown. Conversely, current studies of *Aux*/*IAA* in the auxin signaling pathway have mainly focused on aspects of plant growth and development, but little attention has been paid to understanding the roles of *Aux*/*IAA* in the auxin-mediated response to environmental interactions, such as drought, nutrient deficiency, and other abiotic stresses. In the future, genetic approaches combined with computational modeling approaches will continue to make important contributions to identifying new candidate genes that regulate *Aux*/*IAA*, and a new, broader layer of auxin signaling regulatory networks may be discovered. Apart from its function in *Arabidopsis*, the model plant, our knowledge regarding *Aux*/*IAA* regulation of plant growth and development is very limited, but it is very clear that our examination of these processes in other plants will greatly benefit from the knowledge that is being obtained in model plants.

The article "Aux/IAA Gene Family in Plants: Molecular Structure, Regulation, and Function" was published in 2018. Journal: Int J Mol Sci.

## Figures and Tables

**Figure 1:** Domain architecture of the canonical Aux/IAA proteins. The canonical Aux/IAA proteins consist of four typical domains, namely, Domains I–IV. Domain I contains an “LxLxL” motif, which is called the ethylene response factor (ERF)-associated amphiphilic repression (EAR) motif. Between Domain I and II, a conserved “KR” motif was identified as a rate motif, and a bipartite nuclear localization signal (NLS) was located between the KR motif and Domain II. The “GWPPV” motif in Domain II is a degron, which controls the turnover of Aux/IAA proteins. Domain III and IV together form type I/II Phox and Bem1p (PB1) domains. Domain III comprises β1, β2, and α1, and the conserved “K” residue in β1 has been identified as a type II basic motif of PB1. Domain IV contains three β-sheets (β3–β5) and two α-helices (α2 and α3). One OPCA-like motif in this domain forms the other face of the ePB1 domain, and a conserved “GDVP” motif between β4 and α2 may facilitate electrostatic protein interactions. Another NLS was also observed in this domain [5,44,60].

**Figure 2:** Aux/IAA protein interaction network. The physical protein–protein interactions were obtained from the BioGRID database (v3.4.153, https://thebiogrid.org/) [76] and visualized in Cytoscape (version 3.5.0) [77]. The Aux/IAA, ARF, TPL/TPR and TIR1/AFB proteins were identified first, and the remaining proteins were classified into different functional categories using MapMan software (version 3.0.0) [78].

**Figure 3:** Aux/IAA proteins might be regulated at different levels. PKL, PICKLE; LAX2, LIKE AUXIN RESISTANT 2; GCN5, general control nonderepressible 5; PIF3, PHYTOCHROME INTERACTING FACTOR 3; PIF4, PHYTOCHROME INTERACTING FACTOR 4; PIF5, PHYTOCHROME INTERACTING FACTOR 5; CBF1, C-repeat binding factor 1; DREB2A, dehydration-responsive element binding protein 2A; bZIP11, basic leucine zipper 11; PHYA, PHYTOCHROME A; RGL3, RGA-LIKE3; UBC13, UBIQUITIN-CONJUGATING ENZYME 13; TIR1, TRA NSPORT INHIBITOR RESPONSE 1/AUXIN SIGNALING F-BOX.

**Figure 4:** Summary of the functions of Aux/IAA genes in growth and development processes of *Arabidopsis thaliana* [18,19].

**Table 1:** Genome-wide identification of the Aux/IAA protein family in 32 plant species.

Species	Protein No.	Truncated Protein No.	Complete Protein No.	Reference
*Amborella trichopoda*	16	8 (50%)	8 (50%)	[29]
*Arabidopsis thaliana*	29	11 (38%)	18 (62%)	[19]
*Brachypodium distachyon*	27	8 (30%)	19 (70%)	[29]
*Brassica rapa*	55	18 (33%)	37 (67%)	[46]
*Brassica napus*	119	75 (63%)	44 (37%)	[36]
*Carica papaya*	18	8 (44%)	10 (56%)	[47]
*Cicer arietinum*	22	10 (45%)	12 (55%)	[37]
Citrus	26	3 (12%)	23 (88%)	[33]
*Cucumis sativus*	27	9 (33%)	18 (67%)	[25]
*Eucalyptus grandis*	26	9 (35%)	17 (65%)	[23]
*Glycine max*	63	22 (35%)	41 (65%)	[37]
*Gossypium raimondii*	44	14 (32%)	30 (68%)	[29]
*Marchantia polymorpha*	1	-	1 (100%)	[41,42]
*Medicago truncatula*	17	6 (35%)	11 (65%)	[48]
*Oryza sativa*	31	5 (16%)	26 (84%)	[28]
*Petunia hybrida*	16	-	-	[40]
*Phalaenopsis equestris*	16	8 (50%)	8 (50%)	[29]
*Physcomitrella patens*	3	1 (33%)	2 (67%)	[29]
*Picea abies*	31	23 (74%)	8 (26%)	[29]
*Populus trichocarpa*	35	11 (31%)	24 (69%)	[26]
*Prunus persica*	24	8 (33%)	16 (67%)	[29]
*Ricinus communis*	21	8 (38%)	13 (62%)	[29]
*Selaginella moellendorffii*	9	7 (77%)	2 (22%)	[40]
*Solanum lycopersicum*	26	3 (12%)	23 (88%)	[24]
*Solanum melongena*	16	-	-	[40]
*Solanum tuberosum*	26	5 (19%)	21 (81%)	[34]
*Sorghum bicolor*	26	2 (8%)	24 (92%)	[49]
*Triticum aestivum*	84	34 (40%)	50 (60%)	[50]
*Triticum urartu*	27	-	-	[50]
*Utricularia gibba*	25	7 (28%)	18 (72%)	[29]
*Vitis vinifera*	26	0 (0%)	26 (100%)	[35]
*Zea mays*	34	10 (29%)	24 (71%)	[27]
